The article "The Impact of Standardized Health Education in Patients with Ischemic Stroke on Patient Management Satisfaction and Quality of Clinical Management Services" was retracted in 2023. Reasons: signs of a paper mill; compromised peer review; unreliable results or conclusions.

# The Impact of Standardized Health Education in Patients with Ischemic Stroke on Patient Management Satisfaction and Quality of Clinical Management Services

**DOI:** 10.1155/2022/5698400

**Published:** 2022-09-07

**Authors:** Jing Chen, Lin Xiang

**Affiliations:** ^1^Department of Radiology, The Third People's Hospital of Hubei Province, Wuhan 430030, China; ^2^Department of Neurology, Hubei No. 3 People's Hospital of Jianghan University, Wuhan 430030, China

## Abstract

**Aim:**

Ischemic stroke is a common brain disease, which seriously affects the quality of life of patients. The purpose of this study was to evaluate the impact of the application of standardized health education in ischemic stroke patients on patient management satisfaction and clinical management service quality.

**Methods:**

220 patients with ischemic stroke were chosen for study target. The research objects were randomly divided into control group (*n* = 110) and education group (*n* = 110) by odd even number draw lots. The control group conducted conventional treatment; on the basis of the control group, the education group received standardized health education. The impact of the application of standardized health education in patients with ischemic stroke on patient management satisfaction and clinical management service quality was analyzed.

**Results:**

The number of health error items in the two groups decreased significantly after 2 months and 3 months of treatment, contrast to before admission, and the number of health error items in the education group was lower than that in the control group, and the difference was statistically significant. After 3 months of treatment, the daily activity score increased and the neurological function score decreased in the two groups, and the daily activity score in the education group was higher than that in the control group, and the neurological function score was lower than that in the control group; the difference was statistically significant. The satisfaction scores of patients in the education group in different aspects such as staff working attitude, health management, diet management, and environmental management were higher than those in the control group, and the disparity was obvious.

**Conclusion:**

The application of standardized health education in patients with ischemic stroke has certain clinical value.

## 1. Introduction

Ischemic stroke is a common vascular brain illness with a complex pathogenesis that is significantly associated with environmental, genetic, and acquired genetic factors [1, 2]. Ischemic stroke is a condition in which patient's cerebral arteries are blocked, resulting in a dysfunctional blood supply to the brain, leading to partial brain tissue necrosis, which severely affects the patient's neurological function [3, 4]. The disease usually occurs suddenly. With the continuous evolution of ischemic stroke, patients' nerves are very vulnerable to damage, and its disability rate is high, which will lead to the obstruction of their limb motor ability, the impairment of their visual and auditory abilities, and the decline of their autonomous activity ability and motor ability, which will seriously influence the level of life of living sufferers [5, 6]. At present, intravenous thrombolysis is used to treat patients in clinic, which has good curative effect, but standardized management has not been formed in disease health education [7, 8]. Therefore, we should find a scientific and standardized health education method to carry out health management and education for their diseases, which can take a vital part in the healthy life, ability, and neurological function recovery of patients [9–11]. In this study, obtained in to our hospital, from September 2019 to December 2021, 220 patients with ischemic stroke were selected as the research objects, and the health management education and training program was formulated to explore its application effect. Now it is reported as follows.

The article "The Impact of Standardized Health Education in Patients with Ischemic Stroke on Patient Management Satisfaction and Quality of Clinical Management Services" was retracted in 2023. Reasons: signs of a paper mill; compromised peer review; unreliable results or conclusions.

## 2. Materials and Methods

### 2.1. Study Subjects

220 patients with ischemic stroke who came to the emergency department of our hospital from September 2019 to December 2021 were randomly divided into education group (*n* = 110) and control group (*n* = 110) by odd even number draw lots. During the study period, no suspension or shedding occurred in both groups. There were 52 males and 58 females in the education group. Aged from 24 to 72, the average age was 45.18 ± 5.46 years old. In the control group, there were 50 males and 60 females. Aged from 28 to 74, the average age was 45.74 ± 5.38 years old. There was no difference in general data such as gender and age of patients (*P* > 0.05), which was comparable. According to the diagnostic criteria for acute ischemic stroke in the “Chinese guidelines for the diagnosis and treatment of ischemic stroke 2014” [9] written by Peng et al. [12], the patient has severe coma and no active consciousness.

### 2.2. Inclusion and Exclusion Criteria

This study was approved by the ethics committee of our hospital. Inclusion criteria are as follows: (1) meet the above diagnostic criteria of ischemic stroke, (2) the surgical characteristics are relatively clear, (3) less than 79 years old, (4) surgery can be arranged within 72 hours after admission, and (5) the patient or his family members sign the medical documents and voluntarily participate. Exclusion criteria are as follows: (1) patients with severe autoimmune diseases, (2) those who had cerebral hemorrhage in the past, (3) patients with severe blood system diseases or coagulation dysfunction, (4) patients with malignant tumors, (5) people with mental disorders, and (6) the patient is in a coma.

The article "The Impact of Standardized Health Education in Patients with Ischemic Stroke on Patient Management Satisfaction and Quality of Clinical Management Services" was retracted in 2023. Reasons: signs of a paper mill; compromised peer review; unreliable results or conclusions.

### 2.3. Treatment Regimens

The control group: the patients were dealt with routine treatment, psychological repair activities, appropriate psychological counseling, and relieving the patients' mood, so as to recover quickly. It was suggested that patients should mainly eat light food.

The education group: implement standardized expert education methods for patients, and the contents were as follows:

1. Establish a nursing expert group, the members of which were mainly composed of experienced clinicians and nurses. The members of the group cooperated closely to discuss nursing intervention measures. Make nursing and recuperation plans in time
2. *Condition Monitoring, Dynamic Monitoring of Patients' Recovery Process, and Monitoring of Patients' Indicators*. Timely give feedback about the recovery of the disease, through reexamination and other ways to understand the patient's condition contrasted, and provide patients with a reasonable dietary plan
3. Create a good ward environment. Ventilate the ward regularly, adjust the temperature to 27-32°C, the air humidity should be 60%-70%, and set warning signs in the ward to create a good environment for patients
4. *Admission Nursing*. The admission nursing of patients required the consent of patients and their families. Under the guidance of doctors, the nursing staff carried out admission nursing in strict accordance with the nursing plan
5. *Psychological Repair*. From the perspective of the patient's treatment process, it was inevitable to have negative emotions about the condition. Nursing staff need to appease patients' emotions, timely give feedback about the effect of patients in the treatment stage, and encourage patients to maintain a stable mood
6. Establish a good doctor-patient relationship. When communicating with patients with ischemic stroke, medical staff should reasonably guide patients to communicate with them in combination with patients' emotions, so as to improve patients' enthusiasm for treatment cooperation
7. *Strengthen Self-Management*. Send disease knowledge manuals and precautions to patients with ischemic stroke, so that patients can understand the disease precautions. The goal should be to improve patient management objectives and medical compliance behavior, so as to achieve patient self-management. Each time you visited patients, you should closely communicate with patients about disease precautions, understand patients' medication, explain the relationship between exercise, diet, and glucose metabolism, and strengthen patients' medical compliance behavior
8. Establish the patient's disease management information, including the basic information of the patient's hospitalization, as well as the living ability and the disease management mode. Carry out neurological rehabilitation training and drug treatment for patients, as well as the key points of first aid after stroke
9. *Discharge Education*. A series of common problems for patients discharged from hospital also need patients to carry out education, such as how to carry out disease self-management, self-care program, and scientific diet plan after discharge. Nurses recorded the above knowledge points into videos for patients to read and learn and finally continued to deepen their cognition and understanding of knowledge points, so as to achieve effective health education (Figure 1).

The article "The Impact of Standardized Health Education in Patients with Ischemic Stroke on Patient Management Satisfaction and Quality of Clinical Management Services" was retracted in 2023. Reasons: signs of a paper mill; compromised peer review; unreliable results or conclusions.

### 2.4. Follow-Up

(1) Standardize health education knowledge. Observe and record the health knowledge evaluation form of the two groups of patients, including stroke and treatment and rehabilitation knowledge, and count the relevant scores. (2) Service quality. The recovery status of patients was assessed by daily activity scale (Barthel Index scale) and neurological function rating scale (NIHSS), and their service and treatment were effectively evaluated. Barthel Index scores range from 0 to 100 points. The higher the score, the stronger the ability of daily activities; NIHSS score was 0-42 points. The higher the score, the more serious the nerve defect. (3) Management satisfaction. A self-made questionnaire was used to evaluate the patients' satisfaction with this visit, including the staff's working attitude, health management, food management, and environmental management. The total score of each part was 25 points, and the full score was set to 100 points

### 2.5. Data Analysis

SPSS 22.0 was utilized to evaluate quantitative data, and the assessment sample was normally distributed with equal variance and written as (*x̅*±*s*). The *t*-test of paired samples was utilized for intracategory comparisons, while the *t*-test of independent samples was used for comparison between two categories. And the difference was taken clinically significant at *P* < 0.05.

## 3. Results

### 3.1. Comparison of Two Groups of Health Knowledge Analysis

On admission, there was no significant difference in health knowledge error item score between the two groups (*P* > 0.05). The number of health knowledge error item in the two groups decreased significantly after 2 months and 3 months of treatment compared with that before admission (*P* < 0.05), and the number of health knowledge error item in the education group was lower than that in the control group; the difference was statistically significant (*P* < 0.05), as shown in Table 1.

The article "The Impact of Standardized Health Education in Patients with Ischemic Stroke on Patient Management Satisfaction and Quality of Clinical Management Services" was retracted in 2023. Reasons: signs of a paper mill; compromised peer review; unreliable results or conclusions.

### 3.2. Comparison of Daily Activity and Neurological Function between the Two Groups

At admission, there was no significant difference in the scores of daily activity and neurological function between the two groups (*P* > 0.05). After 3 months of treatment, the scores of daily activity and neurological function of the two groups increased, and the scores of daily activity and neurological function of the education group were higher than those of the control group and lower than those of the control group. The differences were statistically significant (*P* < 0.05), as shown in Table 2.

### 3.3. Analysis of Patients' Satisfaction in the Two Groups

The satisfaction scores of the patients in the education group in different aspects such as staff working attitude, health management, diet management, and environmental management were higher than those in the control group, and the difference was statistically significant (*P* < 0.05), as shown in Table 3.

## 4. Discussion

Ischemic stroke is a common brain disease, whose pathogenesis is closely related to external environment, psychological factors, and self-immunity. Clinically, the symptoms of ischemic stroke are coma, blurred consciousness, language function, and sensory nerve disorders, which may cause severe loss of activity [13–15]. Patients with ischemic stroke are very prone to ischemia, resulting in hypoxic necrosis of neurons in brain tissue, damage to neurons, and irreversible cell death, which will have a huge impact on the patient's neurological function, and the disease develops rapidly. Soon after, the patient has blurred consciousness, which seriously threatens the patient's life and health [16–18]. At present, hyperbaric oxygen therapy is used in clinic, which can effectively delay the patient's condition and effectively control the blood supply to the brain. However, 25% of patients have serious sequelae, patients' neurological function is damaged, and some patients' neurological function recovery is poor, which can effectively improve patients' activity and cognitive function [19]. Standard education is helpful to evaluate the degree of neurological impairment of ischemic stroke and lay a theoretical basis for the diagnosis of early patients.

With the continuous improvement of people's living standards and the improvement of people's dietary structure and lifestyle, the proportion of patients with ischemic stroke will continue to increase. Ischemic stroke is a common brain disease, which seriously affects people's quality of life. Therefore, patients need to take drugs for a long time to inhibit vascular blockage, but the patients' cognitive level of the disease is low and lack of systematic understanding, which affects the patients' life treatment [20, 21]. Especially in the elderly, the cognitive level of patients with ischemic stroke is low, and they do not listen to the advice of medical staff, which is not conducive to disease control. The difficulties in the management of patients with ischemic stroke are the long disease cycle, many complications, patients' emotional instability, and poor drug control effect.

The article "The Impact of Standardized Health Education in Patients with Ischemic Stroke on Patient Management Satisfaction and Quality of Clinical Management Services" was retracted in 2023. Reasons: signs of a paper mill; compromised peer review; unreliable results or conclusions.

The main advantages of the application of standardized health education: dynamically understand the situation of patients and timely monitor various indicators of patients, and medical staff should provide psychological guidance to patients, so as to grasp the basic situation of patients in time, so that patients can actively cooperate with treatment. This study found that the score of daily activity ability of patients in the education group was significantly higher than that in the control group, and the score of neurological function of patients in the education group was significantly lower than that in the control group. It shows that health standardization education can strengthen rehabilitation training for patients through careful, accurate, and standardized operation, so as to reduce patients' neurological function and improve patients' daily activity ability. Meglio et al. [22] have shown that humanistic care for patients with ischemic stroke can effectively improve their quality of life. When carrying out nursing intervention for patients with ischemic stroke, it is necessary to carry out psychological counseling, establish an optimistic attitude, and handle treatment correctly, which will make patients actively cooperate with treatment, build confidence, and make patients actively seek help. Pay a return visit to patients, monitor their condition in real time, and communicate with patients at any time, which is convenient for correcting patients' behavior in time and strengthening exercise and other aspects and will improve patients' health status in time. This study found that the satisfaction scores of patients in the education group were higher than those in the control group in different aspects such as staff work attitude, health management, diet management, and environmental management. Narayan et al. [23] have conducted comprehensive nursing intervention on patients with ischemic stroke and found that the comprehensive nursing intervention group is significantly higher than the control group, and the cognition of the disease is relatively high. This is mainly because patients are optimistic after treatment with standardized education, and actively cooperate with doctors to significantly improve the curative effect and effectively improve the treatment effect of patients [24–26]. Therefore, health standardized education should be carried out in the treatment of patients with ischemic stroke, and psychological counseling and rehabilitation training should be included in the treatment of patients with ischemic stroke. It is beneficial to the recovery of patients. However, there are some shortcomings in this study, such as single center and small sample size, which lead to the limitations of the research results. It is necessary to design a multicenter and large sample study to further verify the test results.

The article "The Impact of Standardized Health Education in Patients with Ischemic Stroke on Patient Management Satisfaction and Quality of Clinical Management Services" was retracted in 2023. Reasons: signs of a paper mill; compromised peer review; unreliable results or conclusions.

## 5. Conclusion

To sum up, in the treatment of ischemic stroke patients with standardized health education, integrating psychological counseling and rehabilitation training into the treatment of ischemic stroke patients will help patients improve their psychology, establish a positive and optimistic attitude, and teach patients to master medical nursing knowledge and self-care methods. Through the scientific guidance of patients' psychology, diet, and environment, the symptoms of patients can be significantly alleviated, which is worthy of clinical promotion.

## Figures and Tables

**Figure 1:** The application of standardized health education in patients with ischemic stroke can improve the ability of daily activities, enhance the repair of neural function, and increase the nursing satisfaction of patients.

**Table 1:** Comparison of the number of wrong items of health knowledge between the two groups (pieces, *x̅*±*s*).

Category	Instances	On admission	Treatment for 2 months	Treatment for 3 months
Education group	110	31.35 ± 3.38	7.37 ± 1.79^▲^	6.34 ± 1.59^▲^
Control group	110	30.34 ± 6.57	12.31 ± 3.57^▲^	11.34 ± 3.98^▲^
*t* value		1.306	12.973	12.236
*P* value		0.194	0.000	0.000

Note: Compared with the same group at admission, ^▲^*P* < 0.05.

**Table 2:** Comparison of daily activity and neurological function between the two groups (points, *x̅*±*s*).

Category	Instances	Daily activity ability		Neurological function score	
		On admission	Treatment for 3 months	On admission	Treatment for 3 months
Education group	110	56.58 ± 9.97	71.82 ± 7.43^▲^	22.13 ± 3.24	12.21 ± 2.19^▲^
Control group	110	55.04 ± 6.70	64.42 ± 6.06^▲^	22.56 ± 3.97	14.43 ± 3.92^▲^
*t* value		1.345	8.095	0.880	5.185
*P* value		0.180	0.000	0.380	0.000

Note: Compared with the same group at admission, ^▲^*P* < 0.05.

The article "The Impact of Standardized Health Education in Patients with Ischemic Stroke on Patient Management Satisfaction and Quality of Clinical Management Services" was retracted in 2023. Reasons: signs of a paper mill; compromised peer review; unreliable results or conclusions.

**Table 3:** Satisfaction of patients in the two groups (points, *x̅*±*s*).

Category	Instances	Staff working attitude	Health management	Diet management	Environmental management
Education group	110	22.08 ± 1.64	23.31 ± 1.05	22.16 ± 1.09	22.82 ± 1.64
Control group	110	20.25 ± 2.38	21.14 ± 1.89	21.01 ± 1.27	20.28 ± 2.36
*t* value		6.640	10.526	7.207	9.270
*P* value		0.000	0.000	0.000	0.000

## Data Availability

The data used to support the findings of this study are available from the corresponding author upon request.
